The article "Application of Machine Learning and Information Coverage Centralized Genetic Method in Safety Management of Football Training" was retracted in 2023. Reasons: signs of a paper mill; suspected computer-generated content; unreliable results or conclusions; concerns about the data.

# Application of Machine Learning and Information Coverage Centralized Genetic Method in Safety Management of Football Training

**DOI:** 10.1155/2022/2432309

**Published:** 2022-07-14

**Authors:** Chao Zhang, Fang Tu

**Affiliations:** ^1^School of Physical Education, Wuchang Institute of Technology, Wuhan, Hubei 430065, China; ^2^Libary, Wuchang Institute of Technology, Wuhan, Hubei 430065, China

## Abstract

In recent years, China's competitive sports have developed rapidly. Among them, football is a sport with high energy consumption, high intensity, strong antagonism, and high speed. As a result, injuries are common in football practice. It is impossible to do adequate football training in order to avoid such incidents. At the moment, football injury incidents are common, severely limiting the full growth of the sport in China. This work investigates the safety management of football training using machine learning and an information coverage-centralized genetic technique. To begin, this article describes in detail the machine learning and information coverage-centralized genetic algorithm, summarizes the classification of machine learning models, and introduces the verification and evaluation process of machine learning models and trusted information coverage models as an important theoretical basis for football training safety management. Then, the genetic algorithm based on information coverage concentration is used in football training to analyze the safety risk of football training and the analysis of training speed type. The results show that the human factor accounts for the highest proportion in football training safety accidents, accounting for 28.75%. In the analysis of football training speed, the average passing time of medium strength accounts for the highest proportion of 39.75%. In football training, in order to ensure the safety of training, the combination of medium strength and high strength can be adopted to avoid training injury.

## 1. Introduction

As the development in the technology sector has been increasing day by day, it is a well-known fact that these developments are made solely to improve life standard of the human being irrespective of the classes. These developments become more and more realistic with the advent or introduction of the artificial intelligence, which has a specific motive that is if it is possible that machine could replace human beings in activity or functions where it is applicable. Additionally, some AI-based systems have the idea that if activity could not be controlled completely by the AI-based machines, then these machines could possibly be used for the assistance purpose and such systems exist throughout the world in various domains such as in medicine, Mycin is an AI-based system to assist doctor in the diagnosis process. In this regard, machine learning approaches are presented further in order to emphasis on how these automatic system could learn from the environments where these are deployed to perform a specific task. These models could be used in different application domains where the training of the football player in order to control various injuries is one such possible application, which is carried out in this article.

Football training is a training of speed and endurance. It is a combination of aerobic and anaerobic sports [1]. Football endurance training can prolong the sports intensity of athletes. In the process of football training, the main training is speed and endurance training, which involves direction change, short-distance sprint, deceleration, ball sports, etc.; the above training damages athletes' bodies in varying degrees, so we should pay attention to the safety management of football training [2]. In this article, machine learning and information coverage-centralized genetic algorithm are used for football training safety management, and the most suitable way for football players is selected for training to reduce physical injury.

Genetic algorithm is a widely used search algorithm, which is mainly used in generating data. Its core is to design fitness function to analyze football player training data and design corresponding fitness function based on it. By analyzing the current football safety facilities, find out the potential safety hazards and analyze the safety risks of football training [3].

The innovations of this research process are as follows: (1) describing in detail the machine learning and information coverage-centralized genetic algorithm used in football training security management, summarizing the classification and process of machine learning model, evaluating and verifying the machine learning model, and establishing a trusted information coverage model. (2) In football training, the genetic algorithm based on information coverage is applied to analyze the current situation of football training safety facilities and judge the situation of football training facilities in China according to the survey results. The results show that only 5%–8% of coaches will check the goal of football training field in advance and also require to wear leg guards during football training.

Summary of the related work, which is relevant and available online in well-known databases, is depicted in the section, which is given as follows. In these summaries, a brief description of the basic idea presented in the article along with pros and cons is reported. In the next section, the genetic algorithm based on machine learning and information coverage set is described in detail where initially, the GA has been explained extensively with examples and supportive mathematical equations where applicable. In the second last section, the application design of genetic algorithms in the safety management of football training with how it could resolve the issue is reported and the results are presented as well. Concluding remarks are presented to end the article with supportive references.

## 2. Related Work

With the rapid development of football and campus sports, more and more countries begin to pay attention to football safety education. While offering football courses, the United States will also offer a health course. Students can improve their physical and mental health and promote their physical and mental health through this course. The course content includes knowledge about training, competition, sports injury safety awareness, and prevention. Vaishnavi experts put forward that the most vulnerable part of football players is the ankle. During training, strength training in the way of one-foot high jump and landing can reduce the risk of fracture and increase bone density [4]. Narizuka et al. select the spatial evaluation to complete the analysis of football game. Since the spatial evaluation directly affects the passing quality or player formation of football players, build a field-weighted spatial evaluation framework based on the current goal [3]. Acevedo et al. analyzed the tear of the distal medial collateral ligament often occurred in the process of football training and competition, determined the grade of ligament tear, formulated a surgical repair scheme, and restored the athletes to the previous competition level and returned to the field after surgical treatment [5]. Szymanek-Pilarczyk studies modern football and analyzes the high-level efficiency and physical fitness of athletes on the pitch. The results show that the exercise intensity can be significantly increased after short-term training [6]. Teixeira et al. studied football team sports and pointed out that training load monitoring is an important evaluation method to control training and football match, so as to evaluate the cumulative training and match load of football [7]. Wu and Wang proposed that football is a major sport in colleges and universities in China. This project is highly antagonistic and can be used to cultivate students' willpower and physical quality. However, students are prone to ligament strain, ankle sprain, wrist sprain, and fall during football training, resulting in students' timidity during football training [8]. The primary principle of the safety aim of football training, according to Zhang scholar, is “health first.” Based on this, we develop realistic learning objectives and curricular objectives to promote students' sports safety awareness [9]. Most football sports injuries, according to Wu specialists, are caused by athletes' lack of safety knowledge and attention to sports injuries. When sports injuries are not appropriately treated or healed, strenuous training causes subsequent injuries again [10]. Zhong and Wan study the special training of campus football. During football training, we should pay attention to preventing students' sports injury, improve students' football skills as much as possible, and improve the safety of students' sports function training by introducing the special training of header [11].

## 3. Genetic Algorithm Based on Machine Learning and Information Coverage Set

As the GA is a sub-branch of the AI, which has developed to make the learning process of the automatically controlled system more robust and nearer to the way human beings utilized for the solution of the problems or carrying out of the activities described or elaborated. For simplicity and applicability, it is divided into various subpart and implementation is also subject to those sections.

### 3.1. Machine Learning Model Classification

Machine learning is the study and analysis of how to use computers to simulate human learning behavior in order to acquire new skills, technologies, and knowledge. It has been used in all walks of life [12]. The establishment of a machine learning model requires three processes, namely, preprocessing data, training model, and validation and evaluation model, as shown in Figure 1.

Preprocessing data, selecting features, and reducing dimension of features are the primary steps in feature engineering. Preprocessing data necessitates the collection and acquisition of associated data first. In machine learning, the upper limit of model prediction is determined by data and data attributes. Machine learning algorithms gather data knowledge in a number of methods in order to get as near to the upper limit as feasible. Therefore, the training model data must be very typical, which will lead to model fitting, especially for classification problems, data in the sample should not be seriously offset, and there should be no difference in the amount of data between different categories, which will affect the prediction effect of the model [13]. In the data obtained by machine learning, some data values do not belong to a certain dimension, and some missing values or redundant information will occur. Data preprocessing is to deal with such problems, which facilitates ideal results in model training.

#### 3.1.1. *K*-Nearest Neighbor

When classifying a set of sample data with fixed labels, *K*-nearest neighbors need to compare and analyze all the features on the data to be classified and the features on the data to be classified, and then extract the sample set and the *K* data with the highest degree of similarity to the samples to be measured. The labels in these data with the most classifications are the outcomes of the classification of the data to be categorized, as illustrated in Figure 2. The data to be categorized are shown in Figure 2 as a white circle. The categorized training data are represented by blue and yellow circles, while the four closest neighbors to the white circle are all light colors, and the data type to be classified is produced by the *K*-nearest neighbors. *K*-Nearest neighbors are known for their ease of use and great accuracy. This model, on the other hand, has a high spatial complexity and a high computational complexity and is quickly perturbed by imbalanced data.

#### 3.1.2. Multilayer Perceptor

Multilayer perception machines are called artificial neural networks, and the basic unit of this model is neurons. A neuron receives a great number of signals but only outputs one. The output signal is amplified by a preset weight before being sent to the neuron. When the weight is greater than the threshold, the neuron is activated, indicating that the neuron's output is 1, and when the weight is lower than the threshold, it is deactivated, indicating that the neuron's output is 0. Multilayer perceptors are made up of three layers: input, output, and concealed. Each layer has a huge number of neurons that are connected by complete connections prior to each layer. Usually, a simple multilayer perception machine has no other layers but only a hidden layer, which is shown in Figure 3.

### 3.2. Validation and Evaluation of Machine Learning Models

To further evaluate and verify the classification effect after the construction of the machine learning model, the *k*-nearest neighbor cross-validation begins to study how to use the validation data to evaluate the model effect [14]. Confusion matrix is a two-row, two-column matrix composed of false-negative, false-positive, true-negative, and true-positive data obtained from validation data. Fuzzy evaluation indexes such as accuracy, accuracy, recall, and *F*-value are obtained based on the confusion matrix.

Accuracy is used to determine the proportion of total samples that are classified accurately. The following are the main calculations:

(1) $$\begin{array}{c} \text{ACC}=\frac{\text{TP}+\text{TN}}{\text{TP}+\text{FP}+\text{TN}+\text{FN}}\text{.} \end{array}$$

Accuracy refers to the number of positive samples in a sample with positive predictions, calculated as follows:

(2) $$\begin{array}{c} P=\frac{\text{TP}}{\text{TP}+\text{FP}}. \end{array}$$

The recall rate is the probability of all positive samples that are predicted accurately in the predicted results. The following is the calculation formula:

(3) $$\begin{array}{c} R=\frac{\text{TP}}{\text{TP}+\text{FN}}. \end{array}$$

The *F*1 value is an important indicator of recall and accuracy. Here is the formula:

(4) $$\begin{array}{c} F1=\frac{2\times P\times R}{P+R}. \end{array}$$

### 3.3. Trusted Information Coverage Model

This article optimizes network coverage performance by designing an ideal node coverage model, in which the trusted information coverage model digs deeply into the spatial characteristics of the sensor variables. Compared with the disc model and the probability model with different prediction accuracy, this model works together to rebuild the field information to extract the information values in the environment variables. Therefore, the trusted information coverage model is selected as the node coverage model.

Assuming that the actual value of a variable at any point in space *x* at time *t* is represented by *z*^*t*^(*x*), the estimated value is represented by ${\hat{Z}}^{t}\left(x\right)$, and the *f*-rebuild function is fixed, as shown below:

(5) $$\begin{array}{c} f:\left\{z^{t}\left(S_{t}\right)s_{i}\in S\left(x\right)\right\}⟶{\hat{z}}^{t}\left(x\right), \end{array}$$

The upper form *S*(*x*) is the set of all sensors in an interval.

Based on the spatial statistics theory, the distance *d*(*x*, *y*) between *x* and *y* spatial points is large, indicating that the spatial correlation of environment variables at these two points is low. Minimizing the $\left|z^{t}\left(x\right)-{\hat{z}}^{t}\left(x\right)\right|$ error, which is a variable in a random unknown distribution, is required for the reconstruction site information. It can be replaced with the root mean square error as follows:

(6) $$\begin{array}{c} \Phi \left(x\right)=\sqrt{\frac{1}{T}\sum_{t=1}^{T}{\left(z^{t}\left(x\right)-{\hat{z}}^{t}\left(x\right)\right)}^{2}}. \end{array}$$

Upper form Φ(*x*), a small environmental variable reconstruction quality assessment at the spatial *x*-point, indicates a higher quality of reconstruction. The random field needs a fixed *f*-reconstruction function. The reliable information in this random field will cover the spatial location point *x*, and the RMSE value at this point will be calculated if it exceeds that used by users in the actual network. *ε*_0_ value is expressed as Φ(*x*) ≤ *ε*_0_. Trusted information can completely cover the spatial area, and all spatial points in the area can be covered by trusted information.

Information collaborative reconstruction is based on spatial information statistics in kriging. For a point *x* in space, ordinary Kriging estimates ${\hat{Z}}^{t}\left(x\right)$ attribute values using weighted average values of measurements on sensor nodes in the reconstructed area *S*(*x*), as follows:

(7) $$\begin{array}{c} {\hat{Z}}^{t}\left(x\right)=\sum_{i=1}^{\left|S\left(x\right)\right|}\lambda_{i}\left(S_{i}\right),s_{i}\in S\left(x\right), \end{array}$$

Upper form *λ*_*i*_ is the interpolation weighting factor, ordinary Kriging has unbiased properties, and the sum of all the accumulated ownership values is 1, as shown below:

(8) $$\begin{array}{c} \sum_{i=1}^{\left|S\left(x\right)\right|}\lambda_{i}=1, \end{array}$$

Compute the RMSE value of the reconstructed point *x* based on the following formula:

(9) $$\begin{array}{c} \Phi \left(x\right)=\sum_{i=1}^{n}\lambda_{i}\gamma \left(S_{i},x\right)+\mu \left(x\right). \end{array}$$

The above formula *μ*(*x*) generates an *n*+1 system of linear Kriging equations with *n*+1 unknowns, *n*=|*S*(*x*)|, for minimizing the Lagrange multiplier, *γ*(*S*_*i*_, *x*). The variable function parameter *a* represents the spatial relationship of a particular physical attribute. Using formula (9) to find out the information in local space *x* to collaboratively rebuild confidence.

## 4. Application Design of Genetic Algorithms in Safety Management of Football Training

### 4.1. Application of Centralized Genetic Algorithms Based on Information Coverage in Football Training

Genetic algorithm is based on the principles of biogenetics, so the similarity between the genetic algorithm and genetic principle is high. During species evolution, recombinant, and probabilistic gene mutations are used to inherit the superior and continuous characteristics of species from generation to generation, thus making the environment more adaptable. The principle of the genetic algorithm is similar. Initialize the population by using genetic operators, and set a termination condition under the fitness function and iteration operation to obtain the optimal solution of the problem.

In order to maximize the smoothness of the route, the genetic algorithm's training path in the football training safety management process should meet the following three conditions [15]: collision-free movement, better obstacle avoidance to achieve the shortest path, shorter distance on two-dimensional plane, and high smoothness factor of the path. The fitness function, which is based on the distance, obstacle, and smoothness functions, is constructed based on the preceding requirements.

The following are barrier function formulas:

(10) $$\begin{array}{c} f_{1}\left(k\right)=\sum_{i=2}^{m}\sum_{j=1}^{n}\frac{Z_{1}{\left(k\right)}_{\left(i,j\right)}}{D_{1}}. \end{array}$$

The upper form *f*_*i*_(*k*) is the fitness function for avoiding obstacles on *k* routes, where *i* is the number of route nodes, *m* is the number, and *j* is the number of obstacles. *Z*_1_(*k*) is the Euclidean distance between the first path node and the *j* obstacles on *k* routes, and *D*_1_ is the Euclidean distance between the initial and target points of football training.

The distance function is used to represent the path length. Usually, a shorter distance saves a lot of time. The following is the formula for calculating the distance function:

(11) $$\begin{array}{c} f_{2}\left(k\right)=\sum_{i-1}^{m-1}\frac{D_{1}}{D_{2}{\left(k\right)}_{\left(i,i+1\right)}}. \end{array}$$

The upper *D*_2_(*k*) is the Euclidean distance from the first node on the *k*-th path to the next *i*+1.

The smoothness function is used for the overall bending degree of the path. Higher smoothness of the path indicates better motion performance of the robot. The following formulas represent the smoothness function:

(12) $$\begin{array}{c} f_{3}\left(k\right)=\sum_{i}^{m-1}\frac{\theta_{1}}{\theta {\left(k\right)}_{\left(i,i+1\right)}}. \end{array}$$

The following *f*(*x*) fitness function calculation formulas are derived from the above derivation:

(13) $$\begin{array}{c} f\left(x\right)=af_{1}\left(x\right)+bf_{2}\left(x\right)+cf_{3}\left(x\right)+d. \end{array}$$

In the following formulations, *A*, *B*, and *C* are all function modulation coefficients, while *d* is a constant. The population fitness function is expressed in the abovementioned genetic method. According to the real problem, the evolutionary algorithm should create and enhance the function. The fitness function in the control algorithm is a critical function; thus, its adequacy has a direct influence on the algorithm's functioning, as well as the inability to discover the best solution.

### 4.2. Safety of Football Training Facilities

Safety facilities are the most important one in the safety management of football training. At the same time, leg protectors and football shoes are also the basic facilities needed for football training [16]. Focus on examining the details that cause injuries during training, so start with a safety check of your training facilities, including the courts, doors, shoes, and leg protectors. This article investigates the current status of safety facilities prevention in a course, and the results are shown in Table 1.

Higher requirements are put forward for the football field in the course of football training. Because the football field needs to complete various kicking, stepping, and shoveling movements, when the football field is too wet or too dry, phenomena such as stepping on the ball, falling, and so on will occur during the football training which will result in serious injury, sprain, and limb injury problems.

According to the data in Table 1, most coaches do not pay much attention to the environmental facilities of the court during football training. Only 52%–61% of coaches check whether there are stones and rubbish on the court before training. The proportion of dry training sites, bare wires, and checking the environmental safety nearby is 30%. Therefore, in the process of football training safety management, attention should be paid to the safety of the field.

Table 2 shows the research data about the goal device. Some schools do not check the assembly of the goal in advance whether it is fixed on the ground or not; only 5%–8% of the coaches can complete the inspection on the goal, indicating that more than 90% of the coaches have not done the relevant inspection before the football training, resulting in a large number of security risks.

Because football training is a demanding exercise, wearing protective legs during practice can help prevent injuries and lessen foot sprains. As a result, during football training safety management, it is vital to verify whether the protective legs are worn in advance to avoid the protective legs being displaced, resulting in the emergence of foreign instructors and fractures during football training. Only 32.64 percent of coaches require students to wear leg guards and 32.64 percent of coaches need appropriate footwear during football practice, according to the data in Table 3.

## 5. Application Analysis of Football Training Safety Management

Safety of the football players especially in the training process is very important, and a robust and effective mechanism for implementation of the safety strategies is demanding, which is carried out in this article.

### 5.1. Safety Risk Analysis of Football Training

This article studies the implementation of the genetic algorithm based on machine learning and information coverage in football training safety management and focuses on the evaluation and assessment of football safety risk [17]. Through the classification of types, the object of study can be divided into *A*, *B*, and *C*. The injury accidents often happened in the process of football training on campus are analyzed, and the football safety accident cases are analyzed and drawn in Figure 4. The object of analysis is represented by the *x*-axis, which is the common accident risk type in football safety risk management. Longitudinal coordinate *Y* is the magnitude of analysis object, the frequency of safety risk accidents in football training.

In Table 4, there are 7 types of injury accidents, which are common in football training. Each type of accident has a corresponding number. The above types of accidents are analyzed according to coaches, students, sports environment, management of training items, equipment, venues, and other factors. The accident probability caused by each factor is different. Table 4 shows the proportion of each type of accident injury, of which the highest proportion is A-1, and the proportion of individual accidents caused by students during training is 28.75%. Secondly, coaches' incidents (A-2) in the process of football training accounted for 26.25%, the lowest proportion was (A-3) coaches, and other human factors caused by unexpected business accidents accounted for 5%.

Based on these data, draw a line chart of the cumulative percentage of football training safety risk, which is shown in Figure 5.

Analyzing the data in Figure 5 reveals the risk variables associated with campus football accidents. The following are the conclusions: each industry's risk management method has a cumulative percentage between 0 and 90%. The primary danger kinds of football training include A-1 student factor, A-2 coach factor, B-2 sports environment, and C-2 training facilities. The others are really incidental. A-3 has the largest cumulative proportion of accidents (100%), followed by B-1 equipment, location, and other variables (91.26%), all of which are secondary risk factors.

### 5.2. Speed Analysis of Football Training

This article is based on machine learning and information coverage-centralized genetic algorithm for football training safety management. During the practical application, this algorithm is used to analyze the speed problem of football training. Speed is an important part of the football training process, which can be used to control the game time by increasing speed. There are 2–4 tactical or excessive pass attacks during football training, and the average attack time is 16.24 s. Attacks at this speed can damage an athlete's body, resulting in training injuries or competition injuries.  Figure 6 shows the practice times of different passing strengths.

The data in Figure 6 show that the average practice time of big, medium, and small force passes is 32.53%, 39.75%, and 27.85%. In the daily training process, the training strength is mainly of medium strength, with a small amount of power. Therefore, in the training process, the appropriate medium strength can be selected for training, to achieve the safety management of football training, to ensure that teammates pass the ball quickly and accurately in the appropriate position, and to speed up the attack [18].

Table 5 shows the proportion of different sports speeds in the process of football training, in which the proportion of fast, medium, and slow sports is 36.24%, 40.35%, and 23.41%, respectively. The data shows that the highest proportion of running speed is medium speed. In the process of daily football training, in order to ensure the accuracy of passing the ball and defend and attack in a short time, the safety management process of football training will focus on medium speed and speed, so as to ensure better catch cooperation between players and avoid damage to the formation.

## 6. Conclusion

Football is the most popular sport in the world. Football training is divided into speed endurance and physical endurance training. The intensity of the training process is high, and the training process will also kick, pass, grab, and intercept the ball. The above actions will produce sports injuries in varying degrees. Therefore, the safety management of football training cannot be ignored. China has established a perfect football training system. In this article, the genetic method of machine learning and information coverage concentration is used to study the safety management of football training. Through the detailed description of machine learning and information coverage concentration genetic algorithm and its application in football training safety management, the analysis of football training safety risk and training speed is deeply studied. The results show that the human factor accounts for the highest proportion of football training safety accidents. The proportion reached 28.75%. When analyzing the speed of football training, the average time of medium strength passing accounted for the highest 39.75%.

## Figures and Tables

**Figure 1:** Basic process of machine learning model.

**Figure 2:** *K*-nearest neighbor classification graph.

**Figure 3:** Multilayer perception map.

**Figure 4:** Schematic diagram of football injury types.

**Figure 5:** Line chart of cumulative percentage of football training risk.

**Figure 6:** Proportion of time for different passing strength exercises.

**Table 1:** Stadium safety inspection results (*N* = 73).

	Inspect		Not checked	
	Number (PCS)	Percentage (%)	Number (PCS)	Percentage (%)
Is there any toxic substance	6	6.86	69	93.24
Are there grooves or depressions	32	45.12	41	55.16
Whether there is garbage on the surface	46	61.65	27	38.24
Are stones stacked on the court	39	52.13	34	47.96
Are there any obvious wires on the court	21	27.5	54	72.83
Is the site wet	18	25.94	55	74.02
Is the site dry	14	17.85	61	82.97
Is it safe near the stadium	29	39.16	46	62.05

**Table 2:** Result table for safety precautions check of goal set (*N* = 73).

	Inspect		Not checked	
	Number (PCS)	Percentage (%)	Number (PCS)	Percentage (%)
Firmness of goal assembly	6	8.23	68	91.82
Is the goal completely fixed on the ground	5	5.52	70	95.26

**Table 3:** Training safety facility prevention questionnaire (*N* = 73).

	Inspect		Not checked	
	Number (PCS)	Percentage (%)	Number (PCS)	Percentage (%)
Do the shoes fit	26	36.13	46	64.42%
Are foot guards worn	24	32.64	51	68.56

**Table 4:** Types of injury accidents in football training.

Accident type code	Accident type
A-1	Accidents caused by students during football training
A-2	Accidents caused by coaches during football training
A-3	Accidents caused by coaches and others other than students
B-1	Accidents caused by equipment, site, and other factors
B-2	Accidents caused by sports environment
C-1	Accidents caused by safety management factors
C-2	Accidents caused by management training materials

**Table 5:** Running speed training time ratio.

	Run fast (%)	Medium speedrunning (%)	Slow running (%)
Mean value	36.24	40.35	23.41

## Data Availability

The datasets used and/or analyzed during the current study are available from the corresponding author upon reasonable request.
